# Secure Patient Authentication Framework in the Healthcare System Using Wireless Medical Sensor Networks

**DOI:** 10.1155/2021/9954089

**Published:** 2021-07-22

**Authors:** Saeed Ullah Jan, Sikandar Ali, Irshad Ahmed Abbasi, Mogeeb A. A. Mosleh, Ahmed Alsanad, Hizbullah Khattak

**Affiliations:** ^1^Department of Computer Science & IT, University of Malakand, Chakdara 18800, Pakistan; ^2^Department of Computer Science and Technology, China University of Petroleum-Beijing, Beijing 102249, China; ^3^Beijing Key Lab of Petroleum Data Mining, China University of Petroleum-Beijing, Beijing 102249, China; ^4^Department of Computer Science, Faculty of Science and Arts at Belgarn, University of Bisha, Sabt Al-Alaya 61985, Saudi Arabia; ^5^Faculty of Engineering and Information Technology, Taiz University, Taiz 6803, Yemen; ^6^STC's Artificial Intelligence Chair, Department of Information Systems, College of Computer and Information Sciences, King Saud University, Riyadh 11543, Saudi Arabia; ^7^Department of Information Technology, Hazara University Mansehra, Mansehra 21130, Khyber Pakhtunkhwa, Pakistan

## Abstract

Biosensor is a means to transmit some physical phenomena, like body temperature, pulse, respiratory rate, electroencephalogram (EEG), electrocardiogram (ECG), and blood pressure. Such transmission is performed via Wireless Medical Sensor Network (WMSN) while diagnosing patients remotely through Internet-of-Medical-Things (IoMT). The sensitive data transmitted through WMSN from IoMT over an insecure channel is vulnerable to several threats and needs proper attention to be secured from adversaries. In contrast to addressing the security of all associated entities involving patient monitoring in the healthcare system or ensuring the integrity, authorization, and nonrepudiation of information over the communication line, no one can guarantee its security without a robust authentication protocol. Therefore, we have proposed a lightweight and robust authentication scheme for the network-enabled healthcare devices (IoMT) that mitigate all the identified weaknesses posed in the recent literature. The proposed protocol's security has been analyzed formally using BAN logic and ProVerif2.02 and informally using pragmatic illustration. Simultaneously, at the end of the paper, the performance analysis result shows a delicate balance of security with performance that is often missing in the current protocols.

## 1. Introduction

A healthy human body is a prerequisite to happiness, mental ease, and calm existence. Such a body ensures a sound and robust mind too. On the other hand, an unhealthy physique necessitates caring, treating, diagnosing, and preventing a human for injury or any other illness collectively termed as a healthcare system. While managing healthcare, sight negligence can upset the whole process and may turn counterproductive. This negligence and the flawed nursing system are an embarrassment for patient monitoring due to the attached modules to the human body and recurrent power supply. Each time replacement of power-source can also create serious risks for the patient's life. To ease the work of the whole team and stop human errors and aid the medical professional in examining a patient for a disease, technology and network-oriented devices (Internet-of-Medical-Things (IoMT)) are used that guarantee an authentic result [1]. IoMT facilitates healthcare personnel over the Internet and a decision control system without human-patient or patient-computer interaction. Such emerging technology needs novel services for grasping the attention of healthcare industries for the remote monitoring of their patients. This remote monitoring will not only minimize the cost of a disease for a layman, but also provide the facility for the maximum diagnosing of a patient in this crowded world [2].

Similarly, the healthcare industries are ever-growing, taking over 20.4bn technological interconnected and network-enabled devices. These devices have communication competencies that remotely collect patient information and send it to medical professionals for examination and treatment recommendations. However, the transmission of such sensitive data (body temperature, oxygen saturation, the glucose level in the blood, respiratory rate, heartbeat/pulse rate, etc.) is performed via an open network channel, vulnerable to several threats. It needs proper attention to make it secure. Security, communication, and computation cost or media consumption are also necessary, so that a doctor may easily recognize hand gestures, blood vessels contraction/relaxation, the flow of message in the neuron, and central nervous system (CNS) response of a patient, etc. Attention is also needed for a robust detection system, different color recognition, and stereo sequence of an image control via media [3].

The data acquisition and processing competencies of scalable and practicable devices/machines, interconnected devices, embedded sensors, and installed software applications that can push data flow for patient monitoring are at peak today. After sensing the patient, data is transmitted to the medical professional with wireless networks named Wireless Medical Sensor Network (WMSN) (WMSN is a type of self-organizing network with multiple or mini-embedded sensors inside the human body to sense physical conditions with wireless connectivity. The working procedure of WMSN is to transport data among different participating entities or in the coverage area. WMSN is the fundamental foundation of Internet-of-Medical-Things (IoMT) that can enhance patients' medical treatment) to practice for the diagnosis and medical care. The mutual authentication and cross-verification of each participating entity for such a sensitive transmission are impossible without a key-agreement protocol. It not only facilitates patients at home but is useful in diagnosing various types of diseases as well. Besides, health experts, too, are assisted in assessing and giving advice. While patients' data and physicians' diagnoses are linked/transferred via an open network channel, slight negligence may not only be detrimental and counterproductive, but will shatter people's trust as well. Therefore, it needs extra care and a renewed approach to tackle the issues [4].

Amin et al. [5] proposed the scheme for communicating patient-sensitive information to the doctor/medical professional for diagnosis, which is vulnerable to man-in-the-middle, privileged insider attacks, and lack of mutual authentication. We proposed an improved, lightweight authentication framework that mitigates these weaknesses. The proposed scheme's security has been analyzed using the BAN logic and Provierif2.02 toolkit with an informal discussion for justification. The evaluation results show that the scheme is lightweight in contrast to the state-of-the-art protocol in recent literature. As such, we recommend the proposed protocol for practical implementation in the healthcare online patient diagnoses environment. The main contributions of the research are as follows:

1. In IoMT, the medical professionals having mobile-device can securely obtain the real-time patient's status for diagnosing
2. The outdated data broadcasting flaw common in prior protocols designed for the healthcare system has been fully addressed in this research work
3. A simple hash cryptographic function and public-private key pair are used for designing the security protocol that is lightweight and balances performance with security for the fast, reliable, consistent, and low-latency Wireless Medical Sensor Network (WMSN)
4. The sensor revocation/reissue phase demonstrates that, upon stolen or misplaced sensor or mobile device at any time, no one can assess the internally stored credentials, which means that the prospective scheme is free of offline/online identity guessing and stolen-verifier attacks
5. The protocol's security has been scrutinized both formally using BAN logic and informally using realistic illustration, showing the protocol's robustness
6. The protocol's scalability, reachability, integrity, and authorization, as well as security features, have been achieved using ProVerif2.02 simulation

### 1.1. System Model

The wireless technology for the healthcare industry and installed applications in network-enabled devices can communicate seamlessly to the proper device via WMSN, which has limited battery capacity and low latency. It offers back-end services, quick and intelligent network features for IoMT in healthcare services delivery, while the embedded sensors in the human body can collect and communicate physical conditions to the gateway node using the said limited featured wireless network, for example, (i) visual sensor for sight checkup, (ii) pressure sensor on examining the breath duration of a patient or stress of central nervous system (CNS) or the lower part of the mouth, (iii) temperature sensor for finding the normal body heat, (iv) oxygen saturation sensor for oxygenated blood monitoring, (v) EEG/ECG/MRI sensor is for heart and other parts checkup, (vi) ventilator sensor to provide oxygen continuously to a patient, and (vii) imaging, treatment, diagnosing, and data analytics, etc.

Figure 1 represents the system model or architecture in this paper having four (04) main participants: online service provider for the healthcare system (Certificate Authority), the gateway node (GW), a set of sensors inside the patient body, and external user (medical professionals). The certificate authority (CA) is a specialized company that provides connectivity, data processing, and real-time problem-solving capabilities. The gateway node (GW) is an essential component of the system. All sensors and mobile devices used by patient/medical professionals must be fitted with a gateway node (GW) and connected with alternative network services such as 5G, 6G, and other wireless communication interfaces. The external user (medical professional) can access a designated sensor (patient monitoring) from some ward/location/area. When a patient is in a specialized region or location, the gateway node (GW) controls data broadcasting and verifies the patient's validity. The identification of illegitimate sensors or patient or mobile device or medical professional in the designated area or location or any place may also be easily recognized due to the capability of the intermediary agent (gateway-node (GW)).

It is noteworthy that the Certificate Authority (CA) is officially a fully trusted entity. Their confidence must be consistent, because the trust deficit may impair the system's reliability. The proposed scheme ensures that the registration center can be fully trusted by the patient/sensor/medical professional and the gateway node (GW). In contrast, any other entity alone may not be fully trusted.

### 1.2. Threat Model

The Dolev and Yao [6] model tells us about an adversary's authority between two communicating bodies through an open network channel. According to this model, all the possibilities with an attacker are as follows:

- An adversary might extract the stored data from the GW memory/sensor/mobile device of a medical professional and verify some credentials
- An adversary might alter, delete, update, corrupt, or inject false information on participants' communication over a public network channel
- Adversaries can also have the capabilities to replay, modify, or delete the beneficial information exchange among the participants over a private channel
- An adversary can also obtain the internal sensitive credentials from a stolen sensor/mobile device of a medical professional or from the memory of misplaced sensor/mobile device of medical professional either by reverse engineering technique or by using some critical tags in offline mode, but cannot do both at the same time

With an adversary, our threat model additionally includes the following possibilities:

1. Privacy Threat
2. Suppose that an adversary uses aircrack-ng software to extract sensor locations and other helpful information from stolen data packets. In that case, they are using airodump-ng software to detect signal strength, filtering it for additional attacks, and disrupting the synergy by utilizing airplay-ng software to deauthenticate it. The attacker also has the chance to disrupt the entire network by transferring disassociation packets frequently to disguise its normal operations.
3. Stolen-Verifier Threat
4. Suppose that an attacker can physically steal the mobile device of a medical professional or sensor used by a patient and vice versa, or if it is misplaced, lost, or destroyed somewhere from a legitimate user, an adversary can attack it in order to obtain access to the information recorded in the sensor's/mobile device's memory. After that, they can reveal the encrypted data and begin authentication with another hospital's gateway node or sensor used by other medical professionals or patients.
5. Traffic Analysis Threat
6. Suppose that an adversary can drill the data from IoMT and control the communication channel traffic of broadcasting information towards the sensors. The traffic also consists of sensitive patient's physical phenomenon packets transferred between a medical professional's sensor/mobile device and a gateway node; after the adversary's forensic, the packets in traffic can reveal sensitive information about the system. The adversary evaluated it to see if it might be used as a threat.
7. Access Control Threat
8. The adversary also can understand the different policies and inject false information in the communication path, which connects the different participants for useful information exchange. They can also gain complete control of the channel by examining the overall system activities.
9. Identity Spoofing Threat
10. An adversary can obtain the identity of a legitimate participant in the system and maliciously spoof/fool the system. If they become successful in getting legitimate participants' identities, they can easily control the communication line for altering, deleting, or injecting false information in it.

### 1.3. General Architecture of the Network Model

As explained earlier, the main participants in the proposed system are Certificate Authority (CA), Gateway Node (GW), Sensor Node (SN), and Medical Professional (Mobile-Device). The general working scenario of the system is as follows:

- Gateway node, sensor node, and a medical professional will first register with the certificate authority
- Intelligent sensors embedded inside the patient's body can sense physical phenomenon and broadcast it towards the gateway node through resource constraint WMSN
- From the gateway node, with the help of WMSN, the data is transmitted toward medical professionals for possible diagnosis

The diagrammatic representation of the proposed framework is shown in Figure 2.

## 2. Literature Review

Advances in technology for IoMT devices to transmit data of the healthcare domain and communicate with one another are increasing rapidly, and its security is a challenging task. Since their interconnectivity is vulnerable to several threats like other network-enabled devices, therefore, it needs to be appropriately authenticated with each other. Recently, Singh et al. [7] proposed a framework for orthopedics patients in the pandemic period of COVID-19. Such a patient is unable to attend the hospital for treatment due to chances of Corona. They demonstrated how the orthopedics' patient could use it for his/her healthcare at home while being remotely connected with the hospital. The connectivity of both patient and doctor with the hospital using cloud computing is mandatory. Cloud computing offers infrastructure in three specific models, i.e., Software as a Service (SaaS), Platform as a Service (PaaS), and Infrastructure as a Service (IaaS). However, the stakeholders' cloud-saved database usage can create security and interoperability issues; therefore, [7] failed to design a dynamic authentication scheme for the participants. Alsubaei et al. [8] proposed an IoMT security assessment software framework for the developers/hospitals. But they failed to express the secure authentication of associated devices for examining a patient. Sanaz et al. [9] presented secure IoT-Based e-Healthcare architecture for patient monitoring. They installed an intelligent gateway among all the participants during patient monitoring. They proposed an authentication protocol that authenticates all the entities, including an embedded sensor inside the patient for sensing patients' data, time, temperature, and location intelligently, and transmits them to the health professional. A certificate-based methodology was adopted for the transport layer to work on Wireless Medical Sensor Networks (WMSNs), having a gateway node, a full-power computer system, and application software.

Subsequently, Lee et al. [10] suggested that a high-speed ICT tool can remotely be diagnosing a patient by monitoring and supervising his/her physical phenomenon, so that treatment costs can be minimized. They stated that the Graphical Processing Unit (GPU) is mandatory to reduce the load on the CPU during patient-sensitive data processing. However, they used simple encryption/decryption functions, which are not insufficient for security, privacy, and parallel computation. Rahimi et al. [11] enhanced the Datagram Transport Layer Security (DTLS) between the gateway nodes, patent, and medical professional. In addition, they stated that there is no need for a certificate for session initiation among the participants. Gope et al. [12, 13] suggested a useful structure for IoMT applications for data collection and interpretation based on privacy-preserving (P2DCA). Their architecture splits an interconnected network of integrated multimedia sensors into several clusters. A Cluster Head (CH) was defined as a bunch responsible for protecting the privacy of member MSNs and collecting data and location coordinates. Later, grouped multimedia data was analyzed on the cloud server using an artificial neural network for counterpropagation to extract meaningful information through segmentation. To integrate the infrastructure with mobile devices and overcome the shortage of medical services, Usman et al. [14] proposed an authentication protocol that mitigates medical resource misuse. A patient used its user's name and password on a mobile device to sign in to the public. It is without a password and identity table in the database. It satisfies specific standard protection criteria like protecting against offline password guessing attacks, replay attacks, impersonation attacks, man-in-middle attacks, and insider attacks. However, during decision-making at any crucial time, strong encrypted, authentic, and digitally signed information might be difficult to access even for a legitimate user and also vulnerable to known-key and forgery attacks.

Moghaddam et al. [15] implemented a client-based user authentication agent to validate client-side user identity; SaaS has been used to validate unregistered machines' authentication. The scalability, efficiency, security, man-in-the-middle attack, brute force attack, and timing attack have been evaluated according to the parameters. However, they used two separate servers for authentication and cryptography, which is the wastage of resources. Because the same can be managed from a single centralized server, this might decrease the overall cost and increase security. Satheesh et al. [16] proposed a framework for security and privacy in the healthcare system. Patient-centric confidential information and access control with an improved method of encryption was considered. A digital signature algorithm (DSA), patient pseudoidentity, and personal sensitive information protection were identified. The researchers addressed an enhanced security model for authentication and authorization to discover a new technique that can build security, privacy, and cross-verification of e-healthcare credentials. Allouzi and Javed [17] suggested a framework for authentication of health care devices called Soter. It offers a range of advanced features, such as trust of medical devices, promoting virtual federations, and a trust circle for customized and dynamic access control policy. It is worth noting that when an adversary can get a patient's login information by calling close to him, he/she can account for a hijacking attack on it. [18–20] proposed a cryptographic-based authentication framework, but such frameworks do not provide a fast and secure authentication mechanism, because the performance and security are unable to match each other. The researchers of [21, 22] designed a robust protocol for WMSN, in which multimedia type message was securely transmitted among peers. Still, the networks have not been fixed during multimedia message transmission and created hurdles for the end-user. Shrestha et al. [23] suggested a privacy-protection authentication scheme for healthcare information systems, in which they used digital signatures.

A blockchain is also a means of security for protecting healthcare system records. In this regard, Mikula and Jacobsen [29] proposed a blockchain-based authentication scheme for a centralized digital system. Their approach was implemented in the healthcare domain, in which fundamental patient data of size 3.8 MB has been executed in 2-3 seconds. Immutable data history has shown slow execution and wastage of resources data concerning patients. Further, Das et al. [30] proposed a dynamic identity-based authentication scheme that can resist forgery attacks, insider attacks, stolen verifier attacks, and guessing attacks. However, their strategy is suffering from a privileged insider attack, as the password and identity are transmitted from the user openly towards the server. Kumari et al. [31] provided high-level protection without reducing cloud/fog computing performance, mostly when IoMT is used, and they named it Fog-based Access Control Model (FACM). A cloud-based approach is applied in either mobile or nonmobile context, operating as an additional layer for fog servers, and can offer personalized access control environment. However, the execution time is related to several inputs. Upon increasing intakes, the model's performance will be degraded and vulnerable to impersonation and parallel session key attacks and lacks mutual authentication.

Finally, Rathore et al. [32] demonstrated a novel multilayer perception model for securely diagnosing diabetic patients. They said that the insulin pump inside a patient that controls blood glucose transmits patient sensitive information via the wireless channel and can easily be compromised. Neural-network-based multilayer security can provide security to the embedded medical device inside the patient. Their study revealed 91% accuracy upon an evaluation of the linear vector machine. However, still, no one can trust its reliability for such a sensitive treatment. Wu et al. [33] used Identity and password for designing a protocol via WMSN and healthcare applications. They said that, to overcome the noted disadvantages in their designed protocol, a novel approach is required. Their scheme attracts the modern healthcare industry, in which a paramedical professional can examine patent data remotely using a mobile device. However, because there are no encryption/decryption functions, their scheme is vulnerable to stolen-verifier attacks and privileged-insider attacks. Some related literature review is comprehensively described in Table 1.

## 3. Review Analysis of Amin et al. Protocol

Amin et al. [5] proposed a scheme for IoMT using WMSN in the healthcare domain. Their protocol consists of four phases, i.e., setup phase, registration phase, login and authentication phase, and password change phase. Each of these phases is described one by one under the following headings; notations used in their scheme and their description are shown in Table 2.

### 3.1. Setup Phase

The registration center (RC) first selects a secrete key *K* for the gateway node (GW) and calculates SK_GW-SN*j*_ = *h*(ID_SN*j*_||*K*). In contrast, *n* is the number of embedded sensors inside the patient's body, and its *j*^th^ value lies between 1 and *n* (1 ≤ *j* ≤ *n*). The collision-free one way-hash cryptographic function is also defined here in this phase of the protocol as h:{0, 1}^*∗*^ ⟶ {0, 1}^l^.

### 3.2. Registration Phase

For user's registration, a legitimate user *U*_*ia*_ provides ID_*ia*_, PW_*ia*_, and computes HPW = *h*(ID_*ia*_ ⊕ PW_*ia*_) and relays {ID_*ia*_, HPW_*ia*_} towards gateway node (GW) via a secure channel. Upon receiving {ID_*ia*_, HPW_*ia*_} message, the GW calculates Reg_*ia*_ = *h*(ID_*ia*_||*R*_*ia*_||HPW_*ia*_), *A*_*ia*_ = HPW_*ia*_, *B*_*ia*_ = *h*(ID_*ia*_||*R*_*ia*_||*K*), *C*_*ia*_ = *B*_*ia*_ ⊕ *h*(ID_*ia*_ ⊕ *R*_*ia*_ ⊕ HPW_*ia*_), and *D*_*ia*_ = *R*_*ia*_ ⊕ *h*(TID^*ia*^||*K*). It stores {TID_*ia*_, *D*_*ia*_} in its database and sends {TID_*ia*_, Reg_*ia*_, *A*_*ia*_, *C*_*ia*_, *h*(·)} towards user *U*_*ia*_ over a secure channel, where the user can also store all these parameters in its memory, while, for a patient's registration, he/she first provides his/her name to the registration center (RC). RC assigns the requisite sensor and sends it to the medical professional for future monitoring, prescription or diagnosis.

### 3.3. Login and Authentication Phase

The login and authentication phase of [5] has been completed in the following steps:

- In this phase of the protocol, the user *U*_*ia*_ provides identity ID_*ia*_ and password PW_*ia*_ using hand-held device (Smart Phone) and computes HPW^*∗*^_*ia*_ = *h*(ID_*ia*_ ⊕ PW_*ia*_), *R*^*∗*^_*ia*_ = *A*_*ia*_ ⊕ HPW_*ia*_, Reg^*∗*^_*ia*_ = *h*(ID_*ia*_‖*R*^*∗*^_*ia*_‖HPW^*∗*^_*ia*_) and confirms Reg^*∗*^_*ia*_? = Reg_*ia*_; if a match occurs, further computation is performed; else, termination message is displayed. It generates an arbitrary number *R*_1_ and computes *B*^*∗*^_*ia*_ = *C*_*ia*_ ⊕ *h*(ID_*ia*_ ⊕ *R*^*∗*^_*ia*_||HPW_*ia*_), CID_*ia*_ = ID_*ia*_ ⊕ *h*(TID_*ia*_||*R*^*∗*^_*ia*_||*T*_1_), *M*_1_ = *h*(ID_*ia*_||*B*^*∗*^_*ia*_||*R*_1_||*T*_1_), *M*_2_ = *h*(*R*_*ia*_||*T*_1_) ⊕ *R*_1_ and relays {TID_*ia*_, ID_*SNj*_, CID_*ia*_, *M*_1_, *M*_2_, *T*_1_} towards gateway node (GW) via a public network channel.
- The gateway node finds TID_*ia*_ in its storage table, extracts *D*_*ia*_, and computes *R*^*∗*^_*ia*_ = *D*_*ia*_ ⊕ *h*(TID_*ia*_||*K*), ID^*∗*^_*ia*_ = CID_*ia*_ ⊕ *h*(TID_*ia*_||*R*^*∗*^_*ia*_||*T*_1_), *B*^*∗*^_*ia*_ = *h*(ID^*∗*^_*ia*_||*R*^*∗*^_*ia*_||*K*), *R*^*∗*^_1_ = *M*_2_ ⊕ *h*(*R*^*∗*^_*ia*_||*T*_1_), and *M*^*∗*^_1_ = *h*(ID^*∗*^_*ia*_||*B*^*∗*^_*ia*_||*R*^*∗*^_1_||*T*_1_) and confirms *M*^*∗*^_1_? = *M*_1_; if not matched, authentication is denied; else, gateway node generates another arbitrary number *R*_2_ and computes SK_GW−SN*ja*_ = *h*(IDS_*Nja*_||*K*), *M*_3_ = *h*(*h*(*h*(ID_*ia*_||*R*^*∗*^_1_||*R*_2_))||S_*K*GW−SN*ja*_||*R*_2_), *M*_4_ = *h*(ID_*ia*_||*R*_1_||*R*_2_) ⊕ SK_GW−SN*ja*_, *M*_5_ = *R*_2_ ⊕ *h*(SK_GW−SN*ja*_) and relays {*M*_3_, *M*_4_, *M*_5_} message towards senor node (SN_*j*_) via a public network channel.
- The SN_*j*_ computes *R*^/^_2_ = *M*_5_ ⊕ *h*(SK_GW−SN*ja*_), *M*^/^_6_ = *M*_4_ ⊕ SK_GW−SN*ja*_, *M*^/^_3_ = *h*(*h*(*M*^/^_6_||1)||SK_GW−SN*ja*_|| *R*^/^_2_) and confirms *M*^/^_3_? = *M*_3_; if matched, sensor node produces a third arbitrary number *R*_3_, calculates SK = *h*(*M*^/^_6_||*R*_2_||*R*_3_), *M*_7_ = *h*(SK||*R*_3_||SK_GW−SN*ja*_), *M*_8_ = *h*(*R*_2_) ⊕ *R*_3_, and sends {*M*_7_, *M*_8_} message towards GW via the same public network channel.
- The GW computes *R*^/^_3_ = *M*_8_ ⊕ *h*(*R*_2_), SK^/^ = *h*(*h*(ID_*ia*_||*R*_1_||*R*_2_)||*R*_2_||*R*^/^_3_), *M*^/^_7_ = *h*(SK^/^||*R*^/^_3_||SK_GW−SN*ja*_) and confirms *M*^/^_7_? = *M*_7_; if matched, it produces a temporary identity TID^/^_*ia*_, calculates *M*_9_ = *R*_2_ ⊕ *h*(ID_*ia*_||*R*_1_), *M*_10_ = *h*(ID_*ia*_||SK^/^||*R*^/^_3_), *M*_11_ = TID^/^_*ia*_ ⊕ *h*(*R*_2_ ⊕ *R*_3_), and transmits {*M*_8_, *M*_9_, *M*_10_, *M*_11_} message towards user over the same insecure channel.
- The user calculates *R*^/^_2_ = *M*_9_ ⊕ *h*(ID_*ia*_||*R*_1_), *R*^*∗*^_3_ = *M*_8_ ⊕ *h*(*R*^*∗*^_2_), TID^/^_*ia*_ = *M*_11_ ⊕ *h*(*R*^*∗*^_2_ ⊕ *R*^*∗*^_3_), SK^*∗*^ = *h*(*h*(ID_*ia*_||*R*_1_s *M*^/^_10_ = *h*(ID_*ia*_||SK^*∗*^||*R*^*∗*^_3_) and confirms *M*^/^_10_? = *M*_10_; if matched, it relays a confirmation acknowledgement message towards GW and modifies TID_*ia*_ to TID^/^_*ia*_, while the gateway node calculates the fresh value *D*^/^_*ia*_ = *R*_*ia*_ ⊕ *h*(TID^/^_*ia*_||*K*) and interchanges {TID_*ia*_, D_*ia*_} with the new calculates values {TID^/^_*ia*_, *D*^/^_*ia*_}.

### 3.4. Password Change Phase

If a legitimate user wishes to change his/her password, the protocol provides password change facility in a secure way. The user provides his/her ID_*ia*_, and PW_*ia*_ the computations performed are HPW_*ia*_ = *h*(ID_*ia*_ ⊕ PW_*ia*_), *R*^*∗*^_*ia*_ = A_*ia*_ ⊕ HPW_*ia*_, Reg^*∗*^_*ia*_= *h* (ID_*ia*_||*R*^*∗*^_*ia*_||HPW^*∗*^_*ia*_) and confirm Reg^*∗*^_*ia*_? = Reg_*ia*_; if not matched, a denied message is displayed on the user's screen; else, the user is asked to enter a new password. Upon receiving the password change message, the user is now able to enter a fresh password PW^new^_*ia*_ of his/her own choice and computes HPW^new^_*ia*_ = *h*(ID_*ia*_ ⊕ PW^new^_*ia*_), Reg^new^_*ia*_ = *h*(ID_*ia*_|| *R*^*∗*^_*ia*_||HPW^new^_*ia*_), *A*^new^_*ia*_ = *R*^*∗*^_*ia*_ ⊕ HPW^new^_*ia*_, *B*_*ia*_ = *h*(ID_*ia*_||*R*_*ia*_||K), *C*^new^_*ia*_ = *B*_*ia*_ ⊕ *h*(ID_*ia*_ ⊕ *R*^*∗*^_*ia*_ ⊕ HPW^new^_*ia*_) and replace {Reg_*ia*_, *A*_*ia*_, *C*_*ia*_} with{Reg^new^_*ia*_, *A*^new^_*ia*_, *C*^new^_*ia*_}.

### 3.5. Cryptanalysis of Scheme [5]

By applying the Dolev and Yao [6] model, we find the following weaknesses in Amin et al. protocol:

1. Masquerade Attack
2. An attacker can quickly identify the secret credentials from CID_*ia*_ = ID_*ia*_ ⊕ *h*(TID_*ia*_ǁ*R*^*∗*^_*ia*_ǁT_1_) and *M*_2_ = *h*(*R*_*ia*_ǁ*T*_1_)*R*_1_. The adversary first recovers ID_*ia*_ from CID_*ia*_, and then *R*_1_ from *M*_2_. These two are crucial parameters, and once an attacker gets access to these, he/she can masquerade the system.
3. Privileged Insider Attack
4. Let a user *U*_*ia*_ transmit identity ID_*ia*_ and password PW_*ia*_ towards gateway-node (GW). The system operator, in which he/they can use the system, can quickly identify user credentials by either guessing password or computing HPW_*ia*_^*∗*^ = *h*(ID_*ia*_ ⊕ PW_*ia*_) and run tuples to correct the password.
5. Man-In-The-Middle Attack
6. In such a scheme, authors do not share the synchronized resource's detail. For example, after a successful login of the medical professional to monitor his/her patient, such scheme missed the secure log out procedure of him/her. According to the given scenario, the mutual authentication and cross-verification key are still stored in the synchronous storage. An attacker can easily copy and launch a man-in-the-middle attack, desynchronizing the shared resources, and can hang the system proper operations.
7. Password Change Phase Issue
8. An attacker can easily initiate a new password request by using the power analysis technique. He/she first reaches TID_*ia*_, Reg_*ia*_, *h*(·), *A*_*ia*_ and *C*_*ia*_ and calculates *A*_*ia*_ ⊕ HPW_*ia*_ and *h*(ID_*ia*_||*R*^*∗*^_*ia*_||HPW^*∗*^_*ia*_) by confirming Reg^*∗*^_*ia*_? = Reg_*ia*_; if matched, he/she can get the message “Enter your new password,” which is, in turn, harmful for the system.
9. Anonymity Violation
10. According to such scheme of [5], the messages are transmitted over insecure channels like {TID_*ia*_, ID_SN*ja*_, CID_*ia*_, *M*_1_, *M*_2_, *T*_1_}, {*M*_3_, *M*_4_, *M*_5_}, {*M*_7_, *M*_8_}, and {*M*_8_, *M*_9_, *M*_10_, *M*_11_} and in such way, an attacker can easily detect the medical professional due to the match of extracted values/random number from *M*_2_, *M*_5_ and *M*_8_, i.e., *R*_1_, *R*_2_, and *R*_3_. These random numbers can be quickly figured out by an adversary, for whom he/she can easily trace the paramedical professional's location. Also, the attacker can disturb privacy and can quickly launch a traceability attack. Therefore, the scheme suffered from traceability attacks and could not withstand the privacy and legitimacy of a user, either patient or paramedical professional. Also, in the Identity, ID_*ia*_ and ID_SN*j*_ are transmitted openly, in which an attacker can easily pick and launch an attack some other time.
11. Traceability Attack
12. According to the scheme, the messages CID_*ia*_ = ID_*ia*_ ⊕ *h*(TID_*ia*_||*R*^*∗*^_*ia*_||*T*_1_), *M*_2_ = *h*(*R*_*ia*_||*T*_1_) ⊕ *R*_1_, *M*_4_ = *h*(ID_*ia*_||*R*_1_||*R*_2_) ⊕ SK_GW−SN*ja*_, *M*_5_ = *R*_2_ ⊕ *h* (SK_GW−SN*ja*_), and *M*_8_ = *h*(*R*_2_) ⊕ *R*_3_ are transmitted over a public network channel openly, in which an adversary can catch and figure out credentials by specifying location by repeatedly monitoring different sessions started by the same user. To prevent the adversary from figuring out any identity or tracing any credentials like the exact location of a legitimate user, it must be transmitted securely or linked with a vigorous session shared key (SK).
13. Mutual Authentication Issue
14. The gateway node computes the session key as SK_GW−SN*ja*_ = *h*(IDS_*Nja*_||*K*), and the sensor node SK = *h*(*M*^/^_6_||*R*_2_||*R*_3_). In the second round, the gateway node computes the shared session as SK^/^ = *h*(*h*(ID_*ia*_||*R*_1_||*R*_2_)||*R*^*∗*^_2_||*R*^/^_3_) and user SK^*∗*^ = *h*(*h*(ID_*ia*_||*R*_1_||*R*^*∗*^_2_)||*R*_2_||*R*^*∗*^_3_), which means that the key between the user and gateway node is computed. Still, the sensor embedded in the patient does not know about the shared session key. Therefore, the scheme is failed to deliver mutual authentication and cross-verification with/of all the participants.
15. Lack of Revocation/Reissue Phases
16. Besides the drawbacks mentioned above, [5] did not explain the expansion/recede of the network by the addition/revocation of a new patient/professional. The scheme has missed explaining sensor/patient revocation/reissue or professional revocation/reassignment phases.

## 4. Proposed Solution

We will use critical public infrastructure to generate dynamic numbers for each session for such a resource deficit environment. The scheme consists of the setup phase, registration phase, key-agreement phase, password change phase, and revocation/reissue phase; each of these is discussed one by one under the following headings:

### 4.1. Setup Phase

Extract a prime *P*, the CA first generates two random numbers *x*, *y* of size 160 bits, compute a secret key *s* = xP, and *l* = sP called a public key, collision-free hash function *H*(·):{0, 1}^*∗*^⟶{0, 1}^l^. Keep (ID_SN*j*_||*s*) in sensor node, *s*, and *l* in gateway-node, which is the key role in the whole system.

### 4.2. Registration Phase

This phase consists of two subphases, including patients' and medical professionals' registration subphases, which are described as follows:

1. Patient's Registration
2. A patient first sends his/her name to the CA. CA allocates the requisite accurately and offers/entitles the services to medical professionals. CA also shares a patient's Identity and assigned sensor information to a medical professional.
3. Professional Registration Phase
4. The user selects identity ID_*ia*_, password PW_*ia*_, nonce N_*ia*_ and computes DPW_*ia*_ = *h*(PW_*ia*_||*N*_*ia*_||ID_*ia*_), DID_*ia*_ = *h*(ID_*ia*_||*N*_*ia*_) and transmits {DPW_*ia*_, DID_*ia*_} to gateway node over a secure channel. The gateway node has already a secret key *s* and computes *A* = *h*(ID_*ia*_||DID_*ia*_||*s*), *B* = *h*(ID_*ia*_||DPW_*ia*_||*s*), *C* = *A* ⊕ *B* and *O*=*C* ⊕ *h*(ID_*gwt*_||*s*). The gateway-node (GW) stores *O* and sends {*A*, *B*, *C*, *h*(·)} towards user over a secure channel and stores all these parameters in its own record too as shown in Figure 3.

### 4.3. Key Agreement Phase

This phase of the proposed protocol is accomplished in the following steps:

- A user provides his/her identity, and password computations performed are HPW^*∗*^ = *h*(ID_*ia*_ ⊕  PW_*ia*_), *A*^*∗*^ = *h*(ID_*ia*_||*s*||HPW), confirms *A*^*∗*^? = *A*; if not found valid, computation stops; else, it generates *R*_1_, *s*^*∗*^ and computes *B*^*∗*^ = *C* ⊕ *h*(ID_*ia*_ ⊕ *A*^*∗*^||HPW^*∗*^), *F* = *B*^*∗*^ ⊕ *h*(*s*^*∗*^||*A*^*∗*^||*T*_1_), *J*_1_ = *h*(ID_*ia*_||*B*^*∗*^||*R*_1_||*T*_1_), *J*_2_ = ID_*ia*_ ⊕ *h*(*s*||*T*_1_) and *L*_1_ = *E*_*l*_(*J*_2_||*R*_1_||*s*^*∗*^). Finally, it relays {ID_SN_, *F*, *L*_1_, *T*_1_} towards gateway node (GW) over public channel.
- Verifies timestamp, *T*_1_, decrypts *L*_1_ using *s* to obtain ID_*ia*_, *R*_1_ and *s*^*∗*^. Next, it extracts *O* from the already stored record in gateway node (GW) and computes *O*^*∗*^ = *k*⊕h(ID_SN_||*s*) and confirms *O*? = *O*^*∗*^; if not matched, computation stops; else, it computes ID^*∗*^_*ia*_ = *F* ⊕ *h*(*l*||*A*^*∗*^||*T*_1_), *B*^*∗*^ = *h*(ID^*∗*^_*ia*_||*A*^*∗*^||*l*), *R*^*∗*^_1_ = *J*_2_ ⊕ *h*(*A*^*∗*^||*T*_1_), *J*_1_^*∗*^ = *h*(ID^*∗*^_*ia*_||*B*^*∗*^||*R*^*∗*^_1_||*T*_1_) and again confirms *J*_1_^*∗*^? = *J*_1_; if not matched, the process terminated; else, it generates *R*_2_ and computes sk = *h*(ID_SN_||*l*), *L*_3_ = *h*(*h*(*h*(ID_*ia*_||*R*^*∗*^_1_||*R*_2_))||ID_SN_||*R*_2_), *L*_4_ = *h*(ID_*ia*_||*R*_1_||*R*_2_) ⊕ sk, *L*_5_ = *R*_2_ ⊕ ID_SN*j*_ and *L*_6_ = *E*_*l*_(ID_SN_||*R*_1_||*R*_2_||*L*_5_). In this step of the login and authentication phase, the gateway node forwards {*L*_3_, *L*_4_, *L*_5_, *L*_6_} message towards sensor over a public network channel.
- Upon receiving the {*L*_4_, *L*_5_, *L*_6_} message, the sensor node first decrypts *L*_6_ using *s* to obtain ID_SN_, *R*_1_, *R*_2_ and *L*_5_ and computes *R*^*∗*^_2_ = *L*_5_ ⊕ sk, *L*_7_ = *L*_4_ ⊕ sk, *L*_8_ = *h*(*h*(*L*_7_||ID_*P*_)||sk||*R*^*∗*^_2_), *L*_3_^/^ = *h*(*h*(*h*(ID_*ia*_||*R*^*∗*^_1_||*R*^*∗*^_2_))||ID_SN_||*R*_2_) and confirms *L*_3_^/^? = *L*_3_; if not matched, termination of the whole process takes place; else, it generates *R*_3_ and computes sk = *h*(*h*(ID_*ia*_||*R*_1_||*R*^*∗*^_2_)||*R*_2_||*R*_3_), *L*_9_ = *h*(sk||*R*_3_||*R*_1_||*R*^*∗*^_2_), and *L*_10_ = ID_*ia*_||*R*^*∗*^_2_||*R*_2_||*R*_3_ and sends {*L*_9_, *L*_10_} to GW over public channel.
- Further, GW computes and calculates *R*^/^_3_ = *L*_9_||*R*_2_, sk^/^ = *h*(*h*(ID_*ia*_||*R*_1_||*R*^*∗*^_2_)||*R*_2_||*R*^/^_3_), *L*_9_^/^ = *h*(sk^/^||*R*^/^_3_||*R*_1_||*R*^*∗*^_2_) and confirms *L*_9_^/^? = *L*_9_; if found not valid, the process becomes terminated; else, it produces l^*∗*^ and calculates *L*_11_ = *E*_*l*_(*h*(ID_*ia*_||*R*_1_) ⊕ *R*_2_), *L*_12_ = *h*(ID_*ia*_||sk^/^||*R*^/^_3_), *L*_13_ = *E*_*k*_(ID_SN_||l^*∗*^||*L*_11_) and transmits {*L*_11_, *L*_12_} towards user over a public network channel.
- The user first decrypts *L*_11_ using *s* to obtain ID_SN*j*_, *R*_3_, *L*_10_ and calculates *R*^/^_2_ = *L*_11_ ⊕ *h*(ID_*ia*_||*R*_1_), *R*^*∗*^_3_ = *L*_10_||*R*^*∗*^_2_, *A*^/^ = *L*_13_||*h*(*R*^*∗*^_2_ ⊕ *R*^*∗*^_3_), sk^*∗*^ = *h*(*h*(ID_*ia*_||*R*_1_||*R*^*∗*^_2_)||*R*_2_||*R*^*∗*^_3_), *L*^/^_11_ = *h*(ID_*ia*_||sk^*∗*^||*R*^*∗*^_3_) and verifies *L*^/^_11_? = *L*_11_ and keeps sk, sk^/^and sk^*∗*^ session shared keys in each peer for secure message transmission among all the participants as shown in Figure 4, while general framework of the system is shown in Figure 5.

### 4.4. Revocation/Reissue Phase

This phase of the protocol is performed between the user's device and gateway node. The following steps are performed in this phase of the protocol.

- The user provides his/her previous identity ID_*ia*_, password PW_*ia*_, selects new identity ID_*ia*_^new^ and computes *A*_1_ = *h*(ID_*ia*_^new^||*R*_1_), *B*_1_ = *O* ⊕ *A*_1_, *C*_1_ = ID_*ia*_ ⊕ *B*_1_ and transmits {ID_*ia*_, ID_*ia*_^new^, *A*_1_, *C*_1_} towards the gateway node over a secure channel.
- Upon receiving the {ID_*ia*_, ID_*ia*_^new^, *A*_1_, *C*_1_} message, the gateway node computes *B*_1_^*∗*^ = *h*(*s*||*l*||*A*_1_), *C*_1_^*∗*^ = ID_*ia*_ ⊕ *B*_1_^*∗*^, and confirms *C*_1_^*∗*^? = *C*_1_; if not hold, the process is terminated; else, it computes: V_1_ = *h*(ID_*ia*_^new^||*A*_1_), *O*_1_ = *B*_1_^*∗*^ ⊕ *A*_1_, *F*_1_ = *E*_*l*_(*A*_1_||*s*||*l*) and stores {*V*_1_, *O*_1_, *F*_1_, *h*(·)} in its database and transmits it also to the medical device over a secure channel. In this regard, the sensor cancels/evokes/reissues that the process has been made successfully.
- Further, if the medical professional desires to evoke/cancel/reenter, CA asks for entering the Identity ID_*ia*_, and password PW_*ia*_ of the medical professional and computes: *W* = *h*(ID_*ia*_ ⊕ PW_*ia*_), *Y* = *h*(ID_*ia*_||*s*||*W*). CA confirms W and Y in its database; if not correct, the process is terminated; else, CA changes the status of a medical professional as inactive. CA also relays the revocation message to the patient to revoke the medical professional's credentials and transmits the changed status back to CA. Finally, CA also updates the gateway node to revoke the specified medical professional.

### 4.5. Password Change Phase

If a user desires to change his/her password, this protocol provides a password change facility to change the old one with a new one securely. The following steps are performed while changing the password:

- The user provides his/her Identity ID_*ia*_, and old password PW_*ia*_ via its mobile device. The computations performed are DPW_*ia*_ = *h*(ID_*ia*_ ⊕ PW_*ia*_), *A* = *h*(DID_*ia*_||*s*^*∗*^||DPW_*ia*_^*∗*^), and confirm *A*^*∗*^? = *A*; if not matched, a denying message will display on the user's screen; else, it computes *h*(ID_*gwt*_||*s*) ⊕ *N*_*ia*_ and *O*? = *O*^*∗*^ and user is asked to enter the new password.
- Upon receiving the password change message, the medical professional is now able to enter a fresh password PW^new^_*ia*_ of his/her own choice, and computes: DPW^new^ = *h*(ID_*ia*_ ⊕ PW^new^_*ia*_), *A*^new^ = *h* (ID_*ia*_||*s*^*∗*^||DPW^new^), *O*^new^ = *A*^*∗*^ ⊕ DPW^new^, *B*^new^ = *h* (ID_*ia*_||*s*||*l*), *C*^new^ = *B*^new^ ⊕ *h*(ID_*ia*_ ⊕ *A*^*∗*^ ⊕ DPW^new^) and replaces {*A*, *O*, *C*} with{*A*^new^, *O*^new^, *C*^new^}.Therefore, the medical professional can easily change his/her password without interacting with the gateway node and the senor, as shown in Figure 6.

## 5. Security Analysis

In this section, the security analysis of the proposed scheme can be performed both formally and informally. The formal security proof will be performed using a BAN logic and ProVerif2.02 and informal operating assumptions. These are discussed as follows:

### 5.1. BAN Logic Proof

The shared session key sk has been computed among the user, gateway node, and sensor node for future communication. This subsection is a result of This subsection is added in order to prove the scheme's robustness using BAN [27]. BAN is a logic of belief, and trust was first introduced by Mike Burrows, Martin Abadi, and Roger Needham called BAN. The BAN's reasoning covers the following major issues:

- Are participants familiar with one another?
- Do they know if the message is fresh?
- Is it possible to be confident that a third party did not simply insert incorrect information into the original message?

Different rules and their description for the proposed protocol are shown as follows:

(1) Message Meaning
According to this rule, embedded sensor (user) and gateway node communication are carried out on a secure secret session key. Suppose the user believes that the broadcasting between sensor and gateway-node is carried out on session private key SK. Both participants see the message *M* encrypted on key *K*. In that case, the user also believes in the freshness of message *M* exchanged between user and gateway-node.
  (1) $$\begin{array}{c} \frac{U_{ia}|\equiv U_{ia}\overset{\text{SK}}{↔}\text{GW},\;⊲{\left\{M\right\}}_{K}}{U_{ia}|\equiv \text{GW}|∼M},\\ \frac{\text{GW}|\equiv \text{ GW}\overset{\text{SK}}{↔}\text{SN},\;⊲{\left\{M\right\}}_{K}}{\text{GW}|\equiv \;\text{SN}|∼\;M}. \end{array}$$
Similar is the case in gateway node (GW); accordingly, if the gateway node believes that the information exchange among GW and SN is performed through a session shared secret key SK, and both participants see the encrypted message *M* via key *K*; then GW believes SN once said message *M*.
(2) Message Integrity
This rule means that if the user believes that the data transmission over session shared key SK towards gateway node (GW), the message *M* decrypted with key *K*, then the user also believes sensor node once said message *M*.
  (2) $$\begin{array}{c} \frac{U_{ia}|\equiv \;\bar{\overset{\text{SK}}{⟶}}\text{GW},⊲{\left\{M\right\}}_{K^{-1}}}{U_{ia}|\equiv \;\text{GW}|∼M},\\ \frac{U_{ia}|\equiv \;U_{ia}\overset{\text{SK}}{\Rightarrow }\text{GW }⊲{\left\{M\right\}}_{Y}}{U_{ia}|\;\equiv \text{GW}|∼M}. \end{array}$$
Similarly, suppose a user believes the user that the data transmission over session shared key SK towards gateway node (GW) sees the encrypted message *M* via key *K*. In that case, the user also believes the gateway node (GW) once said message *M*.
(3) Seeing Message
If GW believes the data transmission towards SN over SK and sees message *M* via key *K*, then GW also believes SN once said message *M*.
  (3) $$\begin{array}{c} \frac{\text{GW}|\equiv \;\bar{\overset{\text{SK}}{⟶}}\text{SN},⊲{\left\{M\right\}}_{K^{-1}}}{\text{GW}\equiv \;\text{SN}|∼\;M},\\ \frac{\text{GW}|\equiv \text{ GW}\overset{\text{SK}}{\Rightarrow }\text{SN }⊲{\left\{M\right\}}_{Y}}{\text{GW}\equiv \;\text{SN}|∼\;M}. \end{array}$$
Similarly, suppose GW believes data transmission towards Sn through session shared key SK and sees message *M* encrypted over key *K*, then GW believes SN once said message *M*.
(4) Message Authorization
User believes data broadcasting towards Sn over SK and sees the decrypted message *M* through key *Y*, then user also believes GW once said message *M*.
  (4) $$\begin{array}{c} \frac{U_{ia}|\equiv \;\overset{\text{SK}}{\Rightarrow }\text{GW }⊲{\left\{M\right\}}_{Y^{-1}}}{U_{ia}|\equiv \;\text{GW}|∼\;M},\\ \frac{\text{GW}|\equiv \;\overset{\text{SK}}{\Rightarrow }\text{SN }⊲{\left\{M\right\}}_{Y^{-1}}}{\text{GW}|\equiv \text{SN}|∼\;M}. \end{array}$$
Similarly, if GW believes data broadcasting towards SN over Sk and sees the decrypted message *M* via key *Y*, then GW also believes SN once said message *M*.
(5) Message Freshness
Suppose the user believes that the message received is fresh and GW once said message *M*, then both user and GW believe that the received message *M* is also fresh.
  (5) $$\begin{array}{c} \frac{U_{ia}|\equiv \neq \left(M\right),\text{GW}|∼M}{U_{ia}|\equiv \;\text{GW}|\equiv \neq M},\\ \frac{\text{GW}|\equiv \neq \left(M\right),\;\text{SN}|∼M}{\text{GW}|\equiv \;\text{SN}|\equiv \neq M}. \end{array}$$
Similarly, GW believes that *M*'s received message is fresh; SN once said message *M* then both GW and SN also believe that the received message *M* is fresh.
(6) Message Belief
Suppose both user and GW believe jurisdiction and encryption over key *K*, then GW believes encryption on message by key *K*.
  (6) $$\begin{array}{c} \frac{U_{ia}|\equiv \;\text{GW}|\Rightarrow \left(M\right),U_{ia}|\equiv \;\text{GW}|\equiv {\left\{M\right\}}_{K}}{GW|\equiv \;{\left\{M\right\}}_{K}},\\ \frac{U_{ia}|\equiv \;\text{SN}|\Rightarrow \left(M\right),U_{ia}|\equiv \;\text{SN}|\equiv {\left\{M\right\}}_{K}}{\;\text{SN}|\equiv \;{\left\{M\right\}}_{K}}. \end{array}$$
Similarly, if both user and SN believe message jurisdiction and message encryption on key *K*, then SN believes encrypted message *M* through key *K*.
(7) Message Hiding
Suppose user and GW jurisdiction over message *M*, and decrypted message *M* via key *K*, then GW believes the decrypted message *M* via key *K*.
  (7) $$\begin{array}{c} \frac{U_{ia}|\equiv \;\text{GW}|\Rightarrow \left(M\right),U_{ia}|\equiv \;\text{GW}|\equiv {\left\{M\right\}}_{K^{-1}}}{\text{GW}|\equiv \;{\left\{M\right\}}_{K^{-1}}},\\ \frac{U_{ia}|\equiv \;\text{SN}|\Rightarrow \left(M\right),U_{ia}|\equiv \;\text{SN}|\equiv {\left\{M\right\}}_{K^{-1}}}{\text{SN}|\equiv \;{\left\{M\right\}}_{K^{-1}}}. \end{array}$$
Similarly, if a user and SN jurisdiction over message *M*, and decrypted message *M* via key *K*, then SN believes the decrypted message *M* via key *K*.
Remark: |≡ *Believes,*$\overset{\text{sk}}{↔}$*Communication through session key,* ⊲ *sees,*$\overset{\text{SK}}{\Rightarrow }$*Jurisdiction, ∼ once said, # freshness, <M>*_*K*_*encryption using K, <M>*_*K*−1_*Description via K and P*/*Q, if P then Q.*

Now, we are using these rules, equations, and definitions for realizing the secure communication between all the participants of the system. These steps are as follows.

Security goals defined for the proposed protocols are as follows:

  Goal1: *U*_*ia*_|≡ GW $\overset{\text{sk}}{↔}$ *U*_*ia*_
  Goal2: *U*_*ia*_|≡ GW|≡ SN $\overset{\text{sk}}{↔}$ *U*_*ia*_
  Goal3: GW|≡ SN $\overset{\text{sk}}{↔}$ *U*_*ia*_
  Goal4: SN|≡ *U*_*ia*_|≡ GW $\overset{\text{sk}}{↔}$ *U*_*ia*_

The idealization form of the communication message of the protocol is given as follows:

  Msg_1_: *U*_*ia*_ ⟶ GW: {ID_SN_, *F*, *L*_1_, *T*_1_}_*l*_
  Msg_2_: GW ⟶ SN: {*L*_3_, *L*_4_, *L*_6_}_*l*_
  Msg_3_: SN ⟶ GW: {*L*_9_, *L*_10_}_*l*_
  Msg_4_: GW ⟶ *U*_*ia*_: {*L*_11_, *L*_12_, *L*_13_}_*l*_

Assumptions stated for the proposed authentication protocol is as follows:

  Asmpt_1_: *U*_*ia*_|≡ ⧣ (*R*_1_)
  Asmpt_2_: GN|≡ ⧣ (*R*_1_, *R*_2_)
  Asmpt_3_: SN|≡ GN $\overset{k}{↔}$ *U*_*ia*_
  Asmpt_4_: GN|≡ SN $\overset{k}{↔}$ *U*_*ia*_
  Asmpt_5_: *U*_*ia*_|≡ SN $\;\overset{\text{sk}=h\left(L_{7}\|R_{2}\|R_{3}\right)}{↔}$ GN
  Asmpt_6_: SN|≡ GW $\overset{\text{SK}=h\left(h\left(ID_{ia}\|R_{1}\|R_{2}\right)\|R_{2}\|R_{3}\right)}{↔}$ *U*_*ia*_
  Asmpt_7_: *U*_*ia*_|≡ GW ⇒ (*s* ⊕ *R*_1_)
  Asmpt_8_: GW|≡ SN ⇒ (*R*_2_||*l*)
  Asmpt_9_: SN|≡ GW ⇒ (*R*_2_ ⊕ *R*_3_)
  Asmpt_8_: GW|≡ *U*_*ia*_ ⇒ (*R*_3_||*l*^*∗*^)
  Take Msg_1_: *U*_*ia*_ ⟶ GW: {ID_SN_, *F*, *L*_1_, *T*_1_}_*l*_ and Msg_2_: GW ⟶ SN: {*L*_3_, *L*_4_, *L*_6_}_*l*_

Sees rules for the proposed authentication protocol are defined as follows:

 
*S*_1_: GW⊲ {ID_SN_, *F*, *L*_1_, *T*_1_}_*l*_ and SN⊲{*L*_3_, *L*_4_, *L*_6_}_*l*_
  As per Asmpt_1_, and Asmpt_3_ it is stated that:
 
*S*_2_: GW|≡ *U*_*ia*_∼ {ID_SN_, *F*, *L*_1_, *T*_1_}_*l*_
  As per Asmpt_1_, *S*_2_, *s*, and *L*_1_
 
*S*_3_: GW|≡SN|≡ {*L*_9_, *L*_10_}_*l*_
  As per Asmpt_7_, *S*_3_, and Jurisdictional rules
  S_4_: GW|≡ {*L*_9_, *L*_10_}_*l*_
  As per Asmpt_5_, *S*_4_, and *sk*
 
*S*_5_: *U*_*ia*_ |≡ GW|≡ SN $\overset{\text{sk}}{↔}$ *U*_*ia*_**G**_**1**_ Realized
  According to Asmpt_7_, S_5_, and *R*_3_
 
*S*_6_: *U*_*ia*_ |≡ GW|≡ SN $\overset{\text{sk}}{↔}$ *U*_*ia*_**G**_**2**_ Realized
  Msg_3_: SN ⟶ GW: {*L*_9_, *L*_10_}_*l*_, GW ⟶ *U*_*ia*_: {*L*_11_, *L*_12_, *L*_13_}_*l*_ and take Msg_3_ and Msg_4_ as
  Msg_3_: SN ⟶ GW: {*L*_9_, *L*_10_}_*l*_ and Msg_4_: GW ⟶ *U*_*ia*_: {*L*_11_, *L*_12_, *L*_13_}_*l*^*∗*^_
  Applying the seeing rules
 
*S*_7_:*U*_*ia*_⊲GW ⟶ *U*_*ia*_: {*L*_9_, *L*_10_}_*R*_3__, *L*_11_, *L*_12_, *L*_13_}_*l*_, so as per *S*_7_, Asmpt_4_, and *L*_9_
 
*S*_8_: *U*_*ia*_|≡GW∼*h*(*s*||*R*_3_||*l*), as per Asmpt_2_, *S*_8_, *s*, and *L*_12_, gets
 
*S*_9_: SN|≡*U*_*ia*_|≡ *h*(ID_*ia*_||sk^/^||*R*^/^_3_)
  As per Asmpt_6_, *S*_9_, and *L*_9_, *L*_10_
 
*S*_10_: *U*_*ia*_|≡{*L*_11_, *L*_12_, *L*_13_}, as per Asmpt_4_, *S*_10_, and sk
 
*S*_11_: *S*|≡ SN $\overset{\text{sk}}{↔}$ *U*_*ia*_**G**_**3**_ Realized
  As per Asmpt_8_, *S*_11_, and Jurisdictional rules
 
*S*_12_: SN|≡ *U*_*ia*_|≡ GW $\overset{\text{sk}}{↔}$ *U*_*ia*_**G**_**4**_ Realized

It means that all the peers successfully authenticate each other and at any stage do not compromise on a session shared secret key (sk).

### 5.2. Proverif2.02 Simulation

In this subsection of the research paper, a widely used software verification toolkit is used to verify the scheme's confidentiality, authorization, authenticity, and reachability. The ProVerif2.02 simulation code is in appendix A of the paper.

### 5.3. Algorithmic Representation (a Formal Security Validation)

It is to mention that the leading entities in the proposed authentication protocol are Certificate Authority (CA), Gateway Node (GW), Sensor Node (SN), and Medical Professional (User). Gateway node, sensor node, and a medical professional will first register with the certificate authority. The intelligent sensors embedded inside the patient's body can transmit data to the gateway node via a wireless medical sensor network. Finally, from the gateway node, with the help of WMSN, the data is transmitted toward medical professionals. The algorithmic overview/representation of the proposed authentication protocol is shown in Algorithm 1.

#### 5.3.1. Privileged Insider Attack

A privileged user, either medical professional or any other administrator cannot extract any credentials for future usage, as each and everything are kept secret from all types of user.

#### 5.3.2. Ensuring Anonymity

The session key is shared securely, and each computation round trip starts from a separate timestamp, in which the other peer verifies before starting of calculation. Similarly, after data transmission, all the credentials are successfully finished due to the log out facility, so no one traces a legitimate user. Therefore, the proposed protocol is ensuring anonymity and resists traceability drawbacks.

#### 5.3.3. Denial-of-Service (DoS) Attack

As each session starts with a separate session key and time threshold, if an attacker, for example, desires to send false requests to any peer for a disturbance, he/she fails to do so, because Identity, password, and random keys are much secured, and peers respond only to authenticated credentials. Such requests are denied by peers and stopped for such unlawful activity. Therefore, the proposed protocol resists the DoS attack.

#### 5.3.4. Sensor Attack

If two different sensors communicate simultaneously, it will not affect each other due to different identities. Also, the two sessions between the sensor and another user will not act.

#### 5.3.5. Mutual Authentication

As each peer computes the session key sk and shares it for future communication, the proposed protocol has no mutual authentication.

#### 5.3.6. Man-in-Middle Attack

The proposed protocol is modified by sensor revocation and patient revocation phases. These phases successfully log out the requisite user from the process; no credentials were left in either sensor or patient memory. This protocol never allows the evoking entity to start synchronization at any stage in the future. Therefore, the protocol resists the main-in-middle attack.

Finally, the researchers have the following recommendations:

- The proposed work can be tested for a deep learning approach for microarray cancer data classification [34]; graphology based handwritten character analysis for human behavior identification [35] and a deep neural network-based screening model for COVID-19-infected patients using chest X-ray images [36].
- Also, the work done in this research can also be practiced/verified for the rapid COVID-19 diagnosis using ensemble deep transfer learning models from chest radiographic images [37], visibility improvement, and mass segmentation of mammogram images using quantile separated histogram equalization with local contrast enhancement [38–40].

## 6. Performance Evaluations

In this section of the paper, the proposed authentication scheme's performance analysis is performed by finding its storage overheads, computation, and communication. We analyze each of these features by considering the findings of previous experiment by [41, 42].

### 6.1. Attacks and Functionalities Comparison Analysis

Subsequently, it can be compared with some recent and prominent protocols like Kumari et al. [31], Rathore et al. [32], Wu et al. [33], and Amin et al. [5]. The result shows that our scheme is more robust than these schemes. It is worth mentioning that ✓ means that the mentioned attack is “Yes” for the said protocol; it cannot resist and cannot violate the mentioned features, whereas ✖ means that the mentioned security feature is “No” for the said protocol and cannot valid for the mentioned attack, security violation, loophole, etc., as shown in Table 3.

### 6.2. Storage-Overheads Analysis and Comparison

In the work done by [41, 42], identity occupies 64 bits of space, password 60 bits, timestamp 56 bits, secret key 60 bits, MD5 512 bits, encryption 192 bits, and decryption also 192 bits of memory space. Therefore, keeping in view these measures/calculations and computations, the storage overhead analysis of the proposed authentication protocol is shown in Table 4. Upon comparing it with Kumari et al. [31], Rathore et al. [32], Wu et al. [33], and Amin et al. [5], it proves different and fundamental security characteristics/objectives that are higher than those of the mentioned protocols. Graphically, the storage overhead analysis is shown in Figure 7.

**Remark 1 .**

Encryption = 192, decryption = 192 bits, identity = 64 bits, random numbers = 64 bits, MD5 = 512 bits, and public key = 64 bits, calculating for the proposed protocol 192 + 192 + 64(3) + 64(5) + 512 + 512 + 56(3) = 384 + 192 + 320 + 512 + 16 8 = 2088

### 6.3. Computation Costs Analysis and Comparison

Comparing the proposed scheme in terms of computation time complexity due to the experiment performed by [41, 42] of collision-free one-way hash(·) and XOR functions, it is demonstrated that the protocol presented in [31] consists of the registration phase of time complexity for the hash, and XOR functions are 4*t*_*h*_ + 1*t*_⊕_; healthcare system upload phase 14*t*_*h*_ + 6*t*_⊕_; patient upload phase 16*t*_*h*_ + 1*t*_⊕_; treatment phase 15*t*_*h*_ + 6*t*_⊕_ and checkup phase 6*t*_*h*_ + 1*t*_⊕_. The computation time complexity of the proposed scheme is slightly higher compared to [5, 31, 33], as shown in Table 5.

The protocol presented by [31] is a minimum one-way hash time, but it has maximum exponential execution time, while the XOR time complexity is negligibly equal to zero. Rathore et al. [32] used Advanced Encryption Standard (AES) of key size 512, in which polynomial-time generated the random keys, so its hash value is minimal compared to the proposed and [5]. Similarly, [5] used an extra round trip during the login and authentication phase, which our scheme does not have. Therefore, our method consists of a simple hash cryptographic function based; here, it does not affect the computation cost, as shown in Figure 8.

## 7. Conclusion and Future Work

In this modern era, the development of a robust certification environment for the healthcare system gains much attention from researchers, because the intelligent sensors, network-enabled devices (IoMT) and pervasive data acquisition, etc., pushed the healthcare industry to facilitate its patients for diagnoses and remote monitoring. Two things to be focused on for such environment, i.e., information authentication and identification authentication, are challenging, because, without solving these issues and challenges, no one can guarantee secure communication. To ensure data integrity, authorization, nonrepudiation, and user legitimacy and adequately tackle information identification, without a robust authentication protocol, it is not possible. Therefore, we have designed improved, lightweight, and robust authentication protocols for IoMT using WMSN. The proposed protocol mitigated all the known flaws noted for [5] and posed in the existing literature. The robustness of the protocol has been verified using a verification toolkit ProVerif2.00 and BAN logic of belief. In contrast, the performance evaluation result shows that the proposed scheme is fast and secure. The comparison analysis section shows that the proposed protocol is lightweight and balanced with security, often missing in several methods.

In the future, researchers plan to design protocols using the cloud, fog, and edge computing using 5G technology. This is ultra-low latency, which may be utilized for ultra-high reliability in examining a patient's physiological and psychosocial conditions. Also, we plan to discuss the COVID-19 patient X-ray image on a metaheuristic model-based deep learning/screening.

## Figures and Tables

**Figure 1:** Network model.

**Figure 2:** Working procedure of the proposed system.

**Figure 3:** Medical professional registration phase

**Figure 4:** Key agreement phase

**Figure 5:** General framework.

**Figure 6:** Password change phase

**Figure 7:** Storage overheads in bits.

**Figure 8:** Computation cost comparison.

**Algorithm 1:** Algorithmic representation of the proposed protocol.

**Table 1:** Comprehensive literature review.

Reference		Technique used	Main contribution	Limitation
[24]	Klonoff	Certificate-based datagram transport layer security (DTLS)	The proposed scheme consists of a secure and efficient end-user authentication and authorization architecture based on the certificate based DTLS handshake, secure end-to-end communication based on session resumption, and full mobility based on interconnected gateways	The authentication is performed in several steps, due to which multiple round trips can degrade the performance of the process. Also, the securities of the said architecture can easily be breached by an attacker

[25]	Borthakur et al.	Access-control determination (ACD) algorithm	This work proposes a fine-grained access control mechanism suitable for various implementation scenarios, including data storage, directories, and file management	The execution time length is associated with the number of the input task. Therefore the performance will be degraded by increasing the number of input tasks

[26]	Dastjerdi and Buyya	BLE bonding process	This paper addressed some of the fundamental problems. In designing, implementing, and deploying an end-to-end healthcare application that leverages the advantages of the fog computing approach	If the number of corresponding ECG devices increases, more storage will be required, and throughput will be reduced

[27]	Engineer et al.	Contextual-based access control (CBAC) technique and role-based access control (RBAC)	The paper suggested service-oriented security architecture in the IoT environment for remote medical services. The proposed framework accommodates dynamic security elements and requirements regarding different kinds of users	The proposed framework reduces sensitive information exposure by applying a security channel and encryption during the transmission of sensitive information between network parts

[9]	Sanaz et al.	Lightweight anonymous authentication protocol	A secure IoT-based healthcare system was proposed using BSN, called BSN-Care, which can efficiently accomplish various security requirements of the BSN-based healthcare	The proposed work can have stolen verifier attack, replay attack, and anonymity issue

[20]	Wang et al.	Machine learning/deep learning	This paper introduces a novel ECG-based biometric authentication approach that utilizes legendre polynomial extraction and MLP classifier for identification and authorization	Lack of standardization, not accommodate changes to the biometric overtime, sample collection phase is influenced by environmental and mental conditions

[28]	Akrivopoulos et al.	Physical unclonable functions (PUFs)	This paper presents a PUF based device authentication protocol capable of authenticating devices without demanding high CPU power from the end devices	No information about the end device is directly stored on the server, requiring an extra layer of security

**Table 2:** Notations and its descriptions.

Symbol	Description
*U*_*ia*_	Medical professional
SN_*ja*_	Sensor node
ID_*ia*_	User's identity
*K*	Gateway secret key
*R*_1_, *R*_2_, *R*_3_	Random numbers
||	Concatenation function
GW	Gateway node
PW_*ia*_	User's password
ID_*SNj*_	Sensor nodes identity
TID_*ia*_	Temporary-identity generated by GW for *U*_*ia*_
*h*(·)	Collision-free hash-operation
⊕	Bitwise XOR operation

**Table 3:** Attacks and functionalities comparison.

Attack description	[31]	[32]	[33]	[5]	Our
Replay attack	✓	✓	✖	✖	✖
Masquerade attack	✓	✖	✓	✓	✖
Privileged insider attack	✖	✖	✖	✓	✖
Man-in-middle attack	✓	✖	✓	✖	✖
Malicious attack	✓	✓	✓	✖	✖
Anonymity violation	✖	✓	✓	✓	✖
Mutual authentication	✓	✖	✓	✓	✓
DoS attack	✖	✓	✖	✓	✖
Offline guessing attack	✓	✓	✖	✓	✖
Impersonation attack	✓	✖	✓	✖	✖
Spoofing attack	✖	✓	✖	✓	✖
Sensor capture attack	✖	✖	✖	✖	✖

**Table 4:** Storage overhead analysis and comparison.

Protocol	Storage overheads in bits
Kumari et al. [31]	2976
Rathore et al. [32]	3978
Wu et al. [33]	3968
Amin et al. [5]	2112
Our	2088

**Table 5:** Computation cost analysis and comparison.

Protocol	[31]	[33]	[5]	Our
Phase↓				
Registration	4*t*_*h*_ + 1*t*_⊕_	3*t*_*h*_ + 2*t*_⊕_	5*t*_*h*_ + 6*t*_⊕_	3*t*_*h*_ + 3*t*_⊕_
Login and authentication	10*t*_*h*_ + 1*t*_⊕_	19*t*_*h*_ + 11*t*_⊕_	35*t*_*h*_ + 22*t*_⊕_	34*t*_*h*_ + 22*t*_⊕_

## Data Availability

The data collected during the data collection phase will be provided upon request to the corresponding authors.

## Appendix

  (^*∗*^---------*CHANNELS*----------^*∗*^)
  free ChSec:channel [private]. (^*∗*^secure channel between Uia and GW)
  free ChPub:channel. (^*∗*^public channel between User, GW and SN)
  (^*∗*^-----------*SESSION SHARED KEYS*-----------^*∗*^)
  free sk:bitstring [private].
  free skdash:bitstring [private].
  free skstr:bitstring [private].
  (^*∗*^-----------*CONSTANTS AND VARIABLES*---------^*∗*^)
  free IDsn:bitstring.
  free IDia:bitstring.
  free IDiadash:bitstring.
  free SN:bitstring [private].
  free GW:bitstring.
  Free Uia:bitstring.
  free k:bitstring.
  free kstr:bitstring.
  free x:bitstring.
  free xstr:bitstring.
  free PWia:bitstring [private].
  free *R*_1_: bitstring.
  free R1str:bitstring.
  free *R*_2_:bitstring.
  free R2str:bitstring.
  free *R*_3_:bitstring.
  free R3str:bitstring.
  free R1dash:bitstring.
  free R2dash:bitstring.
  free R3dash:bitstring.
  free *T*_1_:bitstring.
  (^*∗*^-------*QUERIES*------^*∗*^)
  query attacker(sk).
  query attacker(skdash),
  query attacker(skstr).
  query attacker(x).
  query attacker(xstr).
  query attacker(*R*_1_).
  query attacker(*R*_2_).
  query attacker(*R*_3_).
  query id:bitstring; inj-event(end_SN(IDsn))==>inj-event(start_SN(IDsn)).
  Query id:bitstring; inj-event(end_IDia(IDia))==>inj-event(start_IDia(IDia)).
  (^*∗*^----------*EVENTS*----------^*∗*^)
  event start_Uia(bitstring).
  event end_Uia(bitstring).
  event start_GW(bitstring).
  event end_GW(bitstring).
  event start_SN(bitstring).
  event end_SN(bitstring).
  (^*∗*^----------*REDUCTIONS and FUNCTIONS*----------^*∗*^)
  fun h(bitstring):bitstring.
  fun mult(bitstring, bitstring):bitstring.
  fun con(bitstring, bitstring):bitstring.
  fun xor(bitstring, bitstring):bitstring.
  fun Encsk(bitstring):bitstring.
  fun Encsksn(bitstring):bitstring.
  fun Decsksn(bitstring):bitstring.
  fun Decsksn(bitstring):bitstring.
  fun PBKDF(bitstring):bitstring.
  (^*∗*^----------*EQUATIONS*----------^*∗*^)
  equation forall *u*: bitstring, *v*: bitstring; xor(xor(*u*, *v*), *u*) = *v*.
  (^*∗*^-------------*USER'S PROCESSES*--------------^*∗*^)
  let Uia = 
  event start_Uia(IDia); let HPWstr = *h*(xor(IDia, PWia) in
  let Astr = *h*(concat(IDia, *x*, HPW)) in
  if Astr = *A* then
  let Bstr = xor(h(xor(concat(*C*, IDia, Astr, HPWstr))) in
  let *F* = xor(h(IDia, (concat(xstr, Astr, *T*_1_))) in
  let *J*_1_ = *h*(concat(IDia, Bstr, *R*_1_, *T*_1_)) in
  let *J*_2_ = xor(*h*(concat(xstr, *T*_1_))) in
  let *L*_1_ = Enc(xor(concat(*J*_2_, *R*_1_, xstr)) in
  out(ChPub, (IDsn, *F*, *L*_1_, *T*_1_)); in(ChPub, (*L*_11_: bitstring, *L*_12_: bitstring, *L*_13_: bitstring)); let Dec(concat(IDsn, *k*, *L*_11_)) in
  let R2dash = xor(*L*_11_, *h*(concat(IDia, *R*_1_))) in
  let R3str = concat(*L*_10_, Rstr2)) in
  let Adash = xor(*L*_13_, h(xor(R2str, R3str))) in
  let skstr = *h*(*h*(concat(IDia, *R*_1_, R2str), *R*_2_, R3str)) in
  let L11dash = *h*(concat(IDia, skstr, R3str)) in
  if L11dash = *L*_11_ then
  event end_Uia(IDia)
  else
  0.
  (^*∗*^-------------*SENSOR NODE PROCESSES*--------------^*∗*^)
  let UiaReg = 
  in(ChSec, (IDia:bitstring, HPWia:bitstring)); let HPWia = concat(PWia, Nia) in
  let *A* = *h*(concat(IDia, IDg, *x*)) in
  let *B* = *h*(concat(IDia, HPWia, *x*)) in
  let *C* = xor(*C*, *B*) in
  let *O* = xor(Nia, *h*(concat(IDsn, *x*))) in
  out(CheSec, (*A*, *B*, *C*)); let GW = 
  event start_GW(IDGW); in(ChPub, (IDsn:bitstring, *F*: bitstring, *T*_1_: bitstring)); Dec(concat(*J*_2_, *R*_1_, xstr)) in
  let Ostr = xor(*R*_1_, *h*(concat(IDsn, xstr))) in
  if Ostr = *O* then
  let IDiastr = xor(*F*, *h*(concat(*R*_1_, Astr, *T*_1_))) in
  let Bstr = *h*(concat(IDia, *A*, *R*_1_)) in
  let R1str = xor(*J*_2_, *h*(concat(Astr, *T*_1_))) in
  let J1str = *h*(concat(IDiastr, Bstr, R1str, *T*_1_)) in
  if J1str = *J*_1_ then
  let sk = *h*(concat(IDsn, *R*_1_)) in
  let *L*_3_ = *h*(*h*(*h*(concat(IDia, R1str, *R*_2_, h(concat(IDsn, *R*_2_))))) in
  let L_4_ = xor(*h*(concat(IDia, *R*_1_, *R*_2_), sk)) in
  let *L*_5_ = sor(*R*_2_, IDsn) in
  let *L*_6_ = Enc(concat(IDsn, *R*_1_, *R*_2_, *L*_5_)) in
  out(ChPub, (*L*_3_, *L*_4_, *L*_5_, *L*_6_)); in(ChPub, (*L*_9_: bitstring, *L*_10_: bitstring)); let Dec(concat(IDsn, *R*_1_, *R*_2_), sk)) in
  let R3dash = concat(*L*_9_, *R*_2_)) in
  let skdash = *h*(h(concat(IDia, *R*_1_, R2str), *h*(*R*_2_, R3dash)) in
  let L9dash = *h*(concat(skdash, R3dash, R2str)) in
  if L9dash = *L*_9_ then
  Let *L*_11_ = xor(h(concat(IDia, *R*_1_), *R*_2_)) in
  Let *L*_12_ = *h*(concat(IDia, skdash, R3dash)) in
  let *L*_13_ = Enc(IDsn, kstr, *L*_11_)) in
  out(ChPub, (*L*_11_, *L*_12_, *L*_13_));
  event end_GW(IDGW)
  else
  0.
  process ((!GW) | (!Uia))
  Running the code, the listed results are displayed, which shows that the attacker could not trace the session share key SK for reconstruction and secure from cracking, as shown below.
  (^*∗*^……………………*RESULT*……………………^*∗*^)
  Completing equations...
  -- Query not attacker(sk),
  Completing...
  Starting query not attacker(sk)
  RESULT not attacker(sk) is true.
  -- Query inj-event(end_Ui(id))==> inj-event(start_Ui(id)),
  Completing...
  Starting query inj-event(end_Ui(id))==> inj-event(start_Ui(id))
  RESULT inj-event(end_Ui(id))==> inj-event(start_Ui(id)) is true.
  -- Query inj-event(end_S(id_57))==> inj-event(start_S(id_57)).
  Completing...
  Starting query inj-event(end_S(id_57))==> inj-event(start_S(id_57))
  RESULT inj-event(end_S(id_57))==> inj-event(start_S(id_57)) is true.
